RETRACTED

# Long non-coding RNA AGAP2-AS1, functioning as a competitive endogenous RNA, upregulates ANXA11 expression by sponging miR-16-5p and promotes proliferation and metastasis in hepatocellular carcinoma

**DOI:** 10.1186/s13046-019-1188-x

**Published:** 2019-05-14

**Authors:** Zhikui Liu, Yufeng Wang, Liang Wang, Bowen Yao, Liankang Sun, Runkun Liu, Tianxiang Chen, Yongshen Niu, Kangsheng Tu, Qingguang Liu

**Affiliations:** Department of Hepatobiliary Surgery, The First Affiliated Hospital of Xi’an Jiaotong University, 277 Yanta West Road, Xi’an, 710061 China

**Keywords:** AGAP2-AS1, Hepatocellular carcinoma, miR-16-5p, ANXA11, Proliferation

## Abstract

**Background:**

Accumulating evidence has highlighted the potential role of long non-coding RNAs (lncRNAs) in the biological behaviors of hepatocellular carcinoma (HCC). Here, we elucidated the function and possible molecular mechanisms of the effect of lncRNA-AGAP2-AS1 on the biological behaviors of HCC.

**Methods:**

EdU, Transwell and flow cytometry were used to determine proliferation, migration, invasion and apoptosis of HCC cells in vitro. The subcutaneous tumor model and lung metastasis mouse model in nude mice was established to detect tumor growth and metastasis of HCC in vivo. The direct binding of miR-16-5p to 3’UTR of ANXA11 was confirmed by luciferase reporter assay. The expression of AGAP2-AS1 and miR-16-5p in HCC specimens and cell lines were detected by real-time PCR. The correlation among AGAP2-AS1 and miR-16-5p were disclosed by a dual-luciferase reporter assay, RIP assay and biotin pull-down assay.

**Results:**

Here, we demonstrated that AGAP2-AS1 expression was up-regulated in HCC tissues and cell lines, especially in metastatic and recurrent cases. Gain- and loss-of-function experiments indicated that AGAP2-AS1 promoted cell proliferation, migration, invasion, EMT progression and inhibited apoptosis of HCC cells in vitro and in vivo. Further studies demonstrated that AGAP2-AS1 could function as a competing endogenous RNA (ceRNA) by sponging miR-16-5p in HCC cells. Functionally, gain- and loss-of-function studies showed that miR-16-5p promoted HCC progression and alteration of miR-16-5p abolished the promotive effects of AGAP2-AS1 on HCC cells. Moreover, ANXA11 was identified as direct downstream targets of miR-16-5p in HCC cells, and mediated the functional effects of miR-16-5p and AGAP2-AS1 in HCC, resulting in AKT signaling activation. Clinically, AGAP2-AS1 and miR-16-5p expression were markedly correlated with adverse clinical features and poor prognosis of HCC patients. We showed that hypoxia was responsible for the overexpression of AGAP2-AS1 in HCC. And the promoting effects of hypoxia on metastasis and EMT of HCC cells were reversed by AGAP2-AS1 knockdown.

RETRACTED

**Conclusions:**

Taken together, this research supports the first evidence that AGAP2-AS1 plays an oncogenic role in HCC via AGAP2-AS1/miR-16-5p/ANXA11/AKT axis pathway and represents a promising therapeutic strategy for HCC patients.

**Electronic supplementary material:**

The online version of this article (10.1186/s13046-019-1188-x) contains supplementary material, which is available to authorized users.

## Background

Hepatocellular carcinoma (HCC) is one of the most common malignancies that leading cancer-associated deaths worldwide [1]. Despite current knowledge and scientific advancement in diagnosis and therapeutic modalities, the long-term survival rate of HCC still remains dismal due to high rate of recurrence and distal metastasis [2–4]. Therefore, it’s critical to discover novel molecular mechanisms which is necessary for developing effective therapeutic strategies for treatment in HCC.

Recently, accumulating evidence confirmed that long non-coding RNAs (lncRNAs) and microRNAs (miRNAs), which completely lack or possess limited protein-coding capacity, are identified as important regulators in the progression of cancers [5–7], including HCC [8]. Aberrant lncRNAs expression play critical roles in cancer progression and carcinogenic through a variety of mechanisms ranging from transcriptional levels to post-transcriptional levels [9]. LncRNA AGAP2-AS1, an antisense lncRNA located at 12q14.1, a novel cancer-related lncRNA, was dysregulated in cancers [10]. Upregulated lncRNA AGAP2-AS1 represses LATS2 and KLF2 expression through interacting with EZH2 and LSD1 in non-small-cell lung cancer cells [11], and its overexpression was associated with malignant clinical features and prognosis [12]. Moreover, lncRNA AGAP2-AS1 promotes cell proliferation and invasion in gastric cancer [13]. However, the expression and its function roles of lncRNA AGAP2-AS1 and its underlying molecular mechanisms in HCC still unknown.

Previous studies confirmed that lncRNAs can interact with miRNAs through miRNA recognition components acting as competing endogenous RNAs (ceRNAs) or “RNA sponges” that can sequester these molecules leading to reduce their regulatory effect on target mRNAs [14, 15]. Our group demonstrated that lncRNA CASC2 suppressed epithelial-mesenchymal transition of hepatocellular carcinoma cells through miR-367/FBXW7 axis [8]. MiRNAs always interacts with complementary sequences within the 3′-untranslated region (UTR) of target mRNA to induce mRNA degradation or translational repression [16, 17]. Increasing studies confirmed that miRNAs are involved in various biological processed in HCC [18]. LncRNAs, mRNA transcripts can affect each other by competitively combining with miRNA response sequence to influence post-transcriptional regulation.

RETRACTED

In present study, we first identified a novel oncogenic lncRNA AGAP2-AS1, was up-regulated in HCC tissues and cells, which may serve as an effective prognostic marker for HCC patients. We also confirmed the expression of miR-16-5p and ANXA11 in HCC, and their effects on the biological behavior of HCC in vitro and in vivo. Furthermore, we explore whether AGAP2-AS1 can regulate the expression of ANXA11 by regulating miR-16-5p expression and affect the biological behavior of HCC. Our results suggest that AGAP2-AS1 exerts a critical role in HCC progression and might be a new molecular target for the treatment of HCC.

## Methods

### Patients’ tissues and cell culture

Patients’ tissues and paired adjacent non-tumor tissues were obtained from patients in our hospital after the informed consent were obtained from all patients. All patients didn’t receive any therapy including radiotherapy, chemotherapy or radiofrequency ablation before surgery. The clinicopathological and demographic information of the patients was described in Table 1. The normal immortalized human hepatocyte LO2 and a panel of HCC cells (Hep3B, HCCLM3, Huh7, MHCC-97H and SMMC-7721) (Chinese Academy of Sciences, Shanghai, China) were maintained in DMEM (Invitrogen, Carlsbad, USA) containing 10% FBS (Gibco, GrandIsland, USA) in 37 °C with 5% CO_2_.

**Table 1:** Correlation between the clinicopathologic characteristics and lncRNA AGAP2-AS1 and miR-16-5p expression in HCC (*n* = 137)

Clinical parameters	Cases	Expression level		*P* value	Expression level		*P* value
		AGAP2-AS1^high^ (*n* = 69)	AGAP2-AS1^low^ (*n* = 68)		miR-16-5p^high^ (*n* = 66)	miR-16-5p^low^ (*n* = 71)	
Age(years)							
< 65 years	76	40	36	0.554	35	41	0.579
≥ 65 years	61	29	32		31	30	
Gender							
Male	109	55	54	0.965	53	56	0.836
Female	28	14	14		13	15	
Tumor size (cm)							
<5 cm	108	48	60	0.007*	59	49	0.004*
≥ 5 cm	29	21	8		7	22	
Tumor number							
solitary	119	59	60	0.637	57	62	0.868
multiple	18	10	8		9	9	
Edmondson							
I + II	98	41	57	0.002*	50	48	0.291
III + IV	39	28	11		16	23	
TNM stage							
I + II	110	50	60	0.020*	58	52	0.031*
III + IV	27	19	8		8	19	
Capsular							
Present	93	47	46	0.953	46	47	0.661
Absent	44	22	22		20	24	
Venous invasion							
Present	18	14	4	0.013*	3	15	0.004*
Absent	119	55	64		63	56	
AFP							
<400 ng/ml	36	21	15	0.265	17	19	0.894
≥ 400 ng/ml	101	48	53		49	52	
HBsAg							
positive	123	61	62	0.592	59	64	0.885
negative	14	8	6		7	7	

*HCC* hepatocellular carcinoma, *AFP* alpha-fetoprotein, *TNM* tumor-node-metastasis

*Statistically significant is in bold

RETRACTED

### Quantitative reverse transcriptase polymerase chain reaction (qRT-PCR)

Total RNA from HCC tissues and cells was isolated using TRIzol reagent (Invitrogen, Carlsbad, CA) according to the manufacturer’s protocol. qRT-PCR was conducted as reported previously. qPCR primers were ordered from Genecopoeia (Guangzhou, China) [19, 20].

### Western blot analysis

We separated proteins by SDS–PAGE and transferred proteins to PVDF membranes. Detailed experiment was performed similar to previously reported [21, 22].

### Immunohistochemical staining (IHC)

The sections were dewaxed, dehydrated, and rehydrated. Primary antibody (1:100, Cell Signaling, Danvers, MA, USA) were added to the sections and incubating at 4 °C overnight. Then applying the biotinylated secondary antibodies (Goldenbridge, Zhongshan, China) according to SP-IHC assays. Specific experiment was conducted similar to previously reported [23].

### Luciferase reporter assay

The 3′-UTR sequence of ANXA11, together with a corresponding mutated sequence within the predicted target sites, were synthesized and inserted into the pmiR-GLO dual-luciferase miRNA target expression vector (Promega, Madison, WI, USA). The assays were carried out as described previously [20, 24].

### RNA immunoprecipitation (RIP) assay

The EZ-Magna RIP Kit (Millipore, USA) was applied to conduct the RIP assay according to the product specification. Firstly, cells were collected and lysed in complete RIP lysis buffer. Then, the cell extract was incubated with RIP buffer containing magnetic beads conjugated to a human anti-Ago2 antibody (Millipore, USA). Samples were incubated with proteinase K with shaking to digest proteins and the immunoprecipitated RNA was isolated. Subsequently, the NanoDrop spectrophotometer was used to measure the concentration of RNA, and the purified RNA was subjected to real-time PCR analysis.

### Cell proliferation, cell cycle and apoptosis detection

EdU and apoptosis were carried as described previously [20, 24].

### Cell migration and invasion analyses

Matrigel-uncoated and -coated transwell inserts (8 μm pore size; Millipore) were used to evaluate cell migration and invasion. Briefly, 2 × 10^4^ transfected cells were suspended in 150 μL serum free DMEM medium into the upper chamber, and 700 Μl DMEM medium containing 20% FBS was placed in the lower chamber. After 24 h incubation, cells were fixed in 4% paraformaldehyde for 20 min and stained with 0.1% crystal violet dye for 15 min. The cells on the inner layer were softly removed with a cotton swab and counted at five randomly selected views, and the average cell number per view was calculated.

RETRACTED

### In vivo experiments

4–6 week-old female BALB/c nude mice (Centre of Laboratory Animals, The Medical College of Xi’an Jiaotong University, Xi’an, China) were used to establish the nude mouse xenograft model and the tail veins for the establishments of pulmonary metastatic model. Mice were sacrificed 3 weeks’ post injection and examined microscopically by hematoxylin and eosin (H&E) staining for the development of lung metastatic foci. The tumor volume for each mouse was determined by measuring two of its dimensions and then calculated as tumor volume = length × width × width/2. Animals were housed in cages under standard conditions. The protocols for these animal experiments were approved by the Ethics Review Committee of Xi’an Jiaotong University.

### Statistical analysis

Results are managed as the mean ± SD and analyzed by SPSS software, 16.0 (SPSS, Chicago, USA). The statistical approaches mainly included a two-tailed Student’s t test, a Kaplan–Meier plot, Pearson chi-squared testand so on. Difference with *P* < 0.05 was regard to be significant. Graphs were mainly made by GraphPad Prism 6 (GraphPad, San Diego, USA).

## Results

### LncRNA AGAP2-AS1 was up-regulated in HCC tissues and associated with HCC progression

To determine the expression level of lncRNA AGAP2-AS1 in HCC, we performed qRT-PCR to examine its level in 50 pairs of randomly selected tumor and corresponding adjacent non-tumor tissues. We demonstrated that AGAP2-AS1 expression was significantly overexpressed in HCC tissues compared to adjacent non-tumor tissues (*P* < 0.05, Fig.1a). Similarly, AGAP2-AS1 was statistically significant increased in a panel of HCC cells lines compared with normal hepatic cell line LO2 (P < 0.05, respectively, Fig.1b). Moreover, we explored the expression level in different clinical progression, and we found that AGAP2-AS1 was up-regulated in large tumor size, metastasis, recurrence and high histological grade tissues (*P* < 0.05, Fig.1c). In general, these results indicated that AGAP2-AS1 potentially has a pivotal role in the progression of HCC.

**Fig. 1:** lncRNA AGAP2-AS1 is up-regulated in HCC and correlates with HCC progression. Comparing differences in the expression of AGAP2-AS1 between (**a**) HCC and matched tumor-adjacent tissues and (**b**) HCC cell lines and the immortalized hepatic cell line LO2. **c** The expression of AGAP2-AS1 in large size (≥5 cm), metastatic tumor tissues, recurrent tumor tissues, high histological grade tumor tissues was significantly increased. *P < 0.05, **P < 0.01

### LncRNA AGAP2-AS1 promoted proliferation, migration and invasion and inhibited apoptosis in HCC in vitro and in vivo

To further investigate the functional roles of AGAP2-AS1 in HCC, we transfected Hep3B who had lowest expression of AGAP2-AS1 with functional pcDNA/AGAP2-AS1 and transfected HCCLM3 who had highest AGAP2-AS1 with specific shRNA (*P* < 0.01, respectively, Fig. 2a). Functionally, Edu assays showed that overexpression of AGAP2-AS1 promoted cell proliferation (*P* < 0.05, Fig. 2b). Transwell assays showed the migration and invasion were increased by AGAP2-AS1 overexpression (*P* < 0.05, Fig. 2c, d). Flow cytometry analysis revealed that AGAP2-AS1 up-regulation inhibited apoptosis in Hep3B cells (P < 0.05, Fig. 2e). EMT progression is of great importance for migration and invasion of HCC cells. Therefore, we attempted to explore whether AGAP2-AS1 had positive effects on HCC cells. WB results indicated that the expression of EMT-related epithelial marker E-cadherin was significantly decreased and the mesenchymal marker Vimentin was dramatically increased by AGAP2-AS1 overexpression same with other EMT indicators. (*P* < 0.05, Fig. 2f, Additional file 1: Figure S1). On the other hand, AGAP2-AS1 knockdown inhibited cell proliferation, migration and invasion and promoted apoptosis in HCCLM3 cells (*P* < 0.05, Fig. 2b-f). These observations demonstrated that AGAP2-AS1 play a critical role in promotion of proliferation and EMT-induced invasion of HCC cells in vitro.

RETRACTED

**Fig. 2:** AGAP2-AS1 promotes cell proliferation, migration, invasion, EMT progress and inhibits apoptosis in HCC cells in vitro. **a** Hep3B and HCCLM3 cells that were transfected with corresponding lncRNA vectors were subjected to qRT-PCR for AGAP2-AS1 expression. Overexpression of AGAP2-AS1 promoted cell proliferation (**b**), migration (**c)**, invasion (**d**) and inhibited apoptosis (**e**) in Hep3B cells, while down-regulation of AGAP2-AS1 inhibited cell proliferation (**b**), migration (**c**), invasion (**d**) and promoted apoptosis (**e**) in HCCLM3 cells. **f** Western blot analysis of EMT-related markers expression in the presence and absence of AGAP2-AS1. n = six independent experiments. *P < 0.05, **P < 0.01, ***P < 0.001

To quantify metastatic potential in vivo, we established a lung metastasis model by tail vein injection. We demonstrated that AGAP2-AS1 overexpression in Hep3B cells promoted the lung metastasis while AGAP2-AS1 knockdown reduced the lung metastasis of HCCLM3 cells (Fig. 3a, *P* < 0.05) by microscopic evaluation. Moreover, we examined the metastasis phenotype of those cells and found that lung sections of overexpressed AGAP2-AS1 in fact showed increased Vimentin expression and conversely increased E-cadherin expression (Fig.3b), while AGAP2-AS1 knockdown showed opposite phenomenon (Fig.3b). Additionally, to determine the effect of AGAP2-AS1 on cell growth in vivo, we used the subcutaneous tumor model to confirm that AGAP2-AS1 overexpression significantly promoted tumor growth, while AGAP2-AS1 knockdown inhibited the tumor growth of HCC cells in mice (*P* < 0.05, Fig. 3c, Additional file 2: Figure S2). Moreover, we used Ki67 and TUNEL staining to evaluate the proliferative and apoptotic rate in the xenografted tissues. As expect, AGAP2-AS1 overexpression increased the Ki67 positive staining cells and reduced the number of apoptotic cells (*P* < 0.05, Fig. 3d and e). However, AGAP2-AS1 knockdown inhibited proliferation and induced apoptosis cells in vivo (*P* < 0.05, Fig. 3d and e). Furthermore, we found that E-cadherin expression in AGAP2-AS1 high expressing HCC tissues was lower than that in low expressing cases. Conversely, the expression of Vimentin in the AGAP2-AS1 high expression group was markedly higher than that in low expression group (*P* < 0.05, respectively, Fig. 3f) Taken together, we demonstrated that AGAP2-AS1 promoted tumor growth and metastasis of HCC in vitro and in vivo.

RETRACTED

**Fig. 3:** AGAP2-AS1 promotes tumor growth and metastasis in vivo*.* **a** Representative HE staining of lung metastases in AGAP2-AS1 overexpression or knockdown cells. **b** Immunohistochemistry of E-cadherin and vimentin were showed and compared between tissues of respective AGAP2-AS1 expression level. **c** Tumor growth curve revealed that AGAP2-AS1 overexpression significantly promoted, while AGAP2-AS1 knockdown inhibited tumor growth in vivo*.* Tumor nodules were subjected to immunohistochemical staining for Ki-67 (**d**) and TUNEL (**e**) assays and quantitative analysis. Representative immunostaining and TUNEL assays revealed that AGAP2-AS1 overexpression significantly increased the number of Ki-67 positive cells and inhibited the number of apoptotic cells. However, the percentage of Ki-67 positive cells in tumors arising from the AGAP2-AS1 knockdown group was significantly lower and the percentage of apoptotic cells was significantly higher than that in the negative control group. **e** Immunohistochemistry of E-cadherin and Vimentin were showed and compared between AGAP2-AS1 high expressing HCC tissues and AGAP2-AS1 low expressing cases. *P < 0.05

### LncRNA AGAP2-AS1 inhibits miR-16-5p via direct binding

Increasing evidence confirmed that lncRNAs function as ceRNAs by binding to miRNAs and mechanically liberating the target RNA transcripts [8]. To explore the potential mechanisms of AGAP2-AS1, we used Starbase v2.0 to predict the potential miRNA binding and found a complementary sequence to miR-16-5p (Fig.4a). miR-16-5p expression was remarkably reduced in HCC tissues comparing to corresponding adjacent non-tumor tissues (*P* < 0.05, Fig. 4b). Furthermore, we found that AGAP2-AS1 expression was negatively associated with the expression of miR-16-5p in HCC tissues (*P* < 0.05, Fig. 4c). Notably, miR-16-5p was down-regulated in AGAP2-AS1 overexpressing Hep3B cells, while miR-16-5p was up-regulated in the AGAP2-AS1 knockdown HCCLM3 cells (P < 0.05, Fig. 4d). Then luciferase reporter assays demonstrated that miR-16-5p significantly inhibited the luciferase activity that carried wild type (wt) but not mutant (mt) 3′-UTR of AGAP2-AS1 (*P* < 0.05, Fig. 4e). Additionally, previous studies confirmed that miRNAs exert its function through binding with Ago2, which is a core component of the RNA-induced silencing complex that is required for miRNAs-induced gene silencing, and the targets of miRNAs can be isolated from complex after Ago2 co-immunoprecipitation. Consistently, results of RIP also confirmed that miR-16-5p was a target of AGAP2-AS1 in HCC cells (*P* < 0.05, Fig. 4f). Furthermore, the biotin-labeled pulldown system demonstrated that a significant amount of AGAP2-AS1 and miR-16-5p in the AGAP2-AS1 pulled down pellet which revealed that AGAP2-AS1 could directly interact with miR-16-5p (*P* < 0.05, Fig. 4g). On the other hand, miR-16-5p also regulated AGAP2-AS1 expression in HCC cells (*P* < 0.05, Fig. 4h). In conclusion, we demonstrated that AGAP2-AS1 could directly bind to miR-16-5p in HCC cells and revealed a reciprocal repression of AGAP2-AS1 and miR-16-5p.

RETRACTED

**Fig. 4:** miR-16-5p was a target of AGAP2-AS1 in HCC. **a** Bioinformatics analysis showed that miR-16-5p could directly target 3′-UTR of AGAP2-AS1-wild type (WT). AGAP2-AS1-mutant (Mut) means mutation of binding sites in the 3′-UTR of AGAP2-AS1. **b** The expression of miR-16-5p in tumor tissues was significantly lower than that in adjacent nontumor tissues. **c** Pearson correlation analysis revealed that an obvious negative association between miR-16-5p and AGAP2-AS1 expression in HCC tissues. **d** Real-time PCR showed that AGAP2-AS1 could negatively regulate miR-16-5p expression in HCC cells. **e** Dual luciferase reporter assays showed that miR-16-5p could negatively regulate the luciferase activity of AGAP2-AS1-WT, rather than AGAP2-AS1-Mut. **f** The association between AGAP2-AS1, miR-16-5p and Ago2 was ascertained by analyzing Hep-3B cell lysates using RNA immunoprecipitation with an Ago2 antibody. Real-time PCR was used to detect the AGAP2-AS1 level change in the substrate of RIP assay in miR-16-5p-overexpressing HCC cells. **g** Detection of AGAP2-AS1 using real-time PCR in the sample pulled down by biotinylated AGAP2-AS1 and negative control (NC) probe. Detection of miR-16-5p using real-time PCR in the same sample pulled down by biotinylated AGAP2-AS1 and NC probe. **h** miR-16-5p inversely regulate AGAP2-AS1 expression in HCC cells. *P < 0.05, ***P < 0.001

RETRACTED

### miR-16-5p served as tumor suppressor and reversed AGAP2-AS1 alteration mediated promotion of proliferation, migration, invasion and EMT in HCC

The expression of miR-16-5p was down-regulated in HCC (Fig. 4b). To investigate the miR-16-5p effect on HCC, we detected cell proliferation, migration, invasion and apoptosis of HCC cells after miR-16-5p overexpression or inhibition (P < 0.05, Fig. 5a). As shown in Fig. 5b-f, the cell proliferation, migration, invasion and EMT progress was inhibited and the apoptosis was promoted by miR-16-5p overexpression, while miR-16-5p knockdown increased the cell proliferation, migration, invasion, EMT progress and decreased apoptosis (P < 0.05, Fig. 5b-f, Additional file 3: Figure S3). To determine whether the tumor-promotive effects of AGAP2-AS1 were mediated by miR-16-5p, we transfected miR-16-5p agomir or antagomir to AGAP2-AS1 alteration cells (P < 0.05, Fig. 5g). Co-transfection of AGAP2-AS1 with agomir-16-5p had the strongest inhibitory effect on cell proliferation, migration and invasion, and promoted the apoptosis of HCC (*P* < 0.05, Fig. 5h-l). Moreover, transfection with antagomirmiR-16-5p rescued the inhibitory effect of sh-AGAP2-AS1 on cell proliferation, migration and invasion, and rescued the increased apoptosis induced in the sh-AGAP2-AS1 group (Fig. 5h-l). Based on the above results, we confirmed that miR-16-5p mediate the tumor-promotive effects of AGAP2-AS1 in HCC cells, and alteration of miR-16-5p respectively reversed the effects induced of AGAP2-AS1 in HCC.

**Fig. 5:** miR-16-5p served as tumor suppressor and reversed AGAP2-AS1 alteration mediated promotion of proliferation, migration, invasion and EMT in HCC. **a** HCCLM3 and Hep3B cells that were transfected with corresponding miRNA vectors were subjected to qRT-PCR for miR-16-5p expression. Overexpression of miR-16-5p inhibited cell proliferation (**b**), migration (**c**), invasion (**d**), EMT process (**f**) and promoted apoptosis (**e**) in HCCLM3 cells, while down-regulation of miR-16-5p promoted cell proliferation (**b**), migration (**c**), invasion (**d**), EMT process (**f**) and inhibited apoptosis (**e**) in Hep3B cells. **g** AGAP2-AS1-overexpressing Hep3B cells that were transfected with empty vector (miR-control) or miR-16-5p overexpression vector were subjected to qRT-PCR for miR-16-5p. AGAP2-AS1-suppressive HCCLM3 cells that were transfected with anti-miR-16-5p were subjected to qRT-PCR for miR-16-5p. miR-16-5p restoration abrogated the effects of AGAP2-AS1 overexpression on cell proliferation (**h**), migration (**i**), invasion (**j**), EMT process (**l**) and apoptosis (**k**) of Hep3B cells. miR-16-5p knockdown reversed the suppressive effects of AGAP2-AS1 knockdown in HCCLM3 cells (**h-l**). *P < 0.05, **P < 0.01

RETRACTED

### Clinical significance of AGAP2-AS1 and miR-16-5p for HCC patients

To explore the clinical significance of AGAP2-AS1 and miR-16-5p in HCC, we divided the patients into different subgroups according to the median value as cutoff and analyzed their correlation with clinical characteristic. As shown in Table 1, we found that AGAP2-AS1 overexpression was significantly associated with large tumor size (≥ 5 cm; *P* = 0.007), high histological grade (Edmondson-Steiner grade III + IV; *P* = 0.002), venous infiltration (*P* = 0.013) and advanced tumor stage (TNM stage III + IV; *P* = 0.020). Meanwhile, miR-16-5p underexpression was dramatically correlated with large tumor size (*P* = 0.004), venous infiltration (*P* = 0.004) and advanced tumor stage (*P* = 0.031). These data revealed that aberrant AGAP2-AS1 and miR-16-5p expression was correlated with poor prognostic features of HCC patients. Furthermore, the Kaplan-Meier survival analysis showed that HCC patients with high AGAP2-AS1 group had a poorer overall survival (OS) and disease-free survival (DFS), while miR-16-5p low-expressing patients presented a shorter OS and DFS (*P* < 0.05, respectively, Fig.6a-d). With combination analysis, we demonstrated that patients with high AGAP2-AS1 and low miR-16-5p expression had the worst OS and DFS (*P* < 0.05, respectively, Fig.6e and f). These data suggest that AGAP2-AS1 and miR-16-5p, especially their combination, is a potential and promising predictor for HCC patients’ prognosis.

**Fig. 6:** The prognostic value of AGAP2-AS1 and miR-16-5p for HCC patients. **a** and (**b**) Overall survival and disease-free survival were compared between AGAP2-AS1 high expressing HCC patients and low expressing cases. **c** and (**d**) Overall survival and (**d**) disease-free survival were compared between miR-16-5p high expressing HCC patients and low expressing cases. **e** and (**f**) Overall survival and disease-free survival were compared between four subgroups of HCC patients. For each cohort, subgroups were divided according to the cutoff values of AGAP2-AS1 and miR-16-5p. The cutoff value was determined as the median value of the relative expression of AGAP2-AS1 and miR-16-5p in HCC tissues. **P < 0.01

### ANXA11 was a direct target gene of miR-16-5p

To explore the mechanisms by which miR-16-5p regulates HCC cell growth and metastasis, informatics tools of three miRNA target-prediction programs (TargetScan, miRDB and PicTar) were used to search for the candidate targets and found ANXA11 3’UTR contains the binding sits of miR-16-5p conserved putative (Fig.7a). we performed luciferase reporter assays to confirm that miR-16-5p overexpression inhibited, while miR-16-5p knockdown increased the luciferase activity of wild type (wt) ANXA11 3’UTR but not the mutant (mt) ANXA11 3’UTR (*P* < 0.05, Fig. 7b). Furthermore, miR-16-5p overexpression significantly inhibited the mRNA and protein expression of ANXA11 in HCCLM3 cells (P < 0.05, respectively, Fig. 7c and d). By contrast, the expression of ANXA11 was significantly increased by miR-16-5p knockdown in Hep3B cells (*P* < 0.05, respectively, Fig.7c and d). Moreover, we found the expressions of ANXA11 in the miR-16-5p high-expressing tumors were significantly lower than those in the miR-16-5p low-expressing tumors (P < 0.05, respectively, Fig. 7e, f). Notably, an obvious inverse correlation between the levels of miR-16-5p and ANXA11 mRNA was revealed by Spearman’s correlation analysis in HCC tissues (*P* < 0.05, Fig. 7g). Next, we explored whether AGAP2-AS1 could regulate the expression of ANXA11. Our data showed that AGAP2-AS1 positively regulated ANXA11 expression in HCC cells (*P* < 0.05, respectively, Fig. 7h, i). In addition, western blot demonstrated that ANXA11 was significantly up-regulated in HCC tissues compared with matched non-tumor tissues (*P* < 0.05, Fig.7j) Thus, we concluded that ANXA11 was a direct target of miR-16-5p and positively modulated by AGAP2-AS1 in HCC cells.

RETRACTED

**Fig. 7:** ANXA11 is a direct target of miR-16-5p in HCC cells. (**a**) miR-16-5p and its putative binding sequences in the 3′-UTR of ANXA11. The mutant binding site was generated in the complementary site for the seed region of miR-16-5p. **b** miR-16-5p overexpression significantly suppressed, while miR-16-5p loss increased the luciferase activity that carried wild-type (wt) but not mutant (mt) 3′-UTR of ANXA11. miR-16-5p overexpression reduced the expression of ANXA11 mRNA (**c**) and protein (D) in HCCLM3 cells and miR-16-5p knockdown increased the level of ANXA11 mRNA (**c**) and protein (**d**) in Hep3B cells. **e** and (**f**) The expression of ANXA11 in miR-16-5p high-expressing tumors was significantly lower than that in miR-16-5p low-expressing tumors, as determined by qRT-PCR and immunoblotting. (**g**) An inverse correlation between the levels of miR-16-5p and ANXA11 mRNA was observed in HCC tissues. AGAP2-AS1 overexpression increased the expression of ANXA11 mRNA (**h**) and protein (**i**) in Hep3B cells and AGAP2-AS1 knockdown reduced the level of ANXA11 mRNA (**h**) and protein (**i**) in HCCLM3 cells. **j** Western blot determined the expression of ANXA11 in HCC and matched tumor-adjacent tissues. *P < 0.05

RETRACTED

### Alteration of ANXA11 expression reversed the biological effects of miR-16-5p and AGAP2-AS1 on HCC cells

To investigate whether ANXA11 mediated the biological function of miR-16-5p and AGAP2-AS1 on HCC cells, ANXA11 was respectively restored in miR-16-5p-overexpressing or AGAP2-AS1 knockdown HCCLM3 cells and inhibited by specific siRNA in miR-16-5p-suppressive or AGAP2-AS1 overexpression Hep3B cells (*P* < 0.05, Fig. 8a). ANXA11 restoration rescued the suppressive effects of miR-16-5p-overexpression or AGAP2-AS1-knockdown HCCLM3 cells on cell proliferation, migration, invasion, apoptosis and EMT progress (P < 0.05, Fig. 8b-f, Additional file 4: Figure S4). Moreover, ANXA11 knockdown abolished the promotive effects of miR-16-5p knockdown or AGAP2-AS1 overexpression Hep3B cells on cell proliferation, migration, invasion, apoptosis and EMT progress (*P* < 0.05, Fig. 8b-f). These results confirm that ANXA11 are functional mediators of AGAP2-AS1/miR-16-5p axis in HCC cells.

**Fig. 8:** Modulation of ANXA11 partially abolishes AGAP2-AS1 or miR-16-5p-mediated cellular processes in HCC. **a** miR-16-5p-overexpressing or AGAP2-AS1-suppressive HCCLM3 cells that were transfected with empty vector (EV) or ANXA11 overexpression plasmid were subjected to western blot for ANXA11. miR-16-5p-suppressive or AGAP2-AS1-overexpressing Hep3B cells that were transfected with scrambled siRNA or ANXA11 siRNA were subjected to western blot for ANXA11. ANXA11 restoration abrogated the effects of miR-16-5p overexpression or AGAP2-AS1 knockdown on cell proliferation (**b**), migration (**c**), invasion (**d**), apoptosis (**e**) and EMT process (**f**) of HCCLM3 cells. ANXA11 knockdown reversed the promotive effects of miR-16-5p knockdown or AGAP2-AS1 overexpression in Hep3B cells (**b-f**). *P < 0.05

### AKT phosphorylation is critical for the biological effects of downstream of ANXA11 in HCC cells

Previous study demonstrated that ANXA11 exerts its function by activating AKT phosphorylation in different cancers [25, 26]. To confirm that AKT phosphorylation mediated the lncRNA AGAP2-AS1/miR-16-5p/ANXA11 axis biological function, we first confirmed that ANXA11 overexpression significantly increased, while ANXA11 knockdown decreased the phosphorylated AKT in HCC cells (*P* < 0.05, respectively, Fig. 9a). To confirm that AKT phosphorylation mediated the effects of ANXA11 on HCC cells, we used AKT inhibitor MK2206 or AKT activator IGF-1 (insulin-like growth factor 1) to alter AKT activation. AKT phosphorylation inhibition by MK2206 in ANXA11-overexpressing Hep3B cells significantly decreased cell proliferation, migration, invasion, EMT progress and induced apoptosis (*P* < 0.05, Fig. 9b-f, Additional file 5: Figure S5). In addition, AKT phosphorylation activator, IGF-1, increased cell proliferation, migration, invasion, EMT progress and inhibited apoptosis (*P* < 0.05, respectively, Fig. 9b-f) in HCCLM3 ANXA11 knockdown cells. Taken together, our results demonstrate that AKT phosphorylation exerts an important role in ANXA11-mediated HCC progression.

RETRACTED

**Fig. 9:** AKT phosphorylation is essential for the biological function of ANXA11 in HCC. **a** HCCLM3 and Hep3B cells that were transfected with corresponding ANXA11 vectors were subjected to immunoblotting for phosphorylated AKT and AKT. AKT inhibitor MK2206, or AKT phosphorylation activator IGF-1, abolished the cell proliferation (**b**), migration (**c**), invasion (**d**), apoptosis (**e**) and EMT process (**f**) of HCC cells which were transduced of ANXA11 vectors. *P < 0.05

### lncRNA AGAP2-AS1 is up-regulated by hypoxia and mediate the promoting effects of hypoxia on HCC cells

After confirming the functional effects and clinical significance of AGAP2-AS1 up-regulation in HCC, we further explored the cause-induced for the increased expression of AGAP2-AS1 in HCC. Previous studies demonstrated that hypoxia is a prevalent tumor microenvironment as a result of an imbalance between oxygen supply and consumption in rapidly growing tumor and plays a critical role in cancer progression. Notably, miR-16-5p, a direct downstream target of AGAP2-AS1 in this study, could be regulated by hypoxia [27, 28]. Therefore, we investigated whether the expression of AGAP2-AS2 could be affected by hypoxia. Hypoxia condition significantly increased HIF-1α expression in Hep3B cells (*P* < 0.05, Fig. 10a) and led to an increase of AGAP2-AS1 expression (*P* < 0.05, Fig. 10b). Interestingly, AGAP2-AS1 knockdown abolished the promoting effects of hypoxia on migration and invasion of Hep3B cells (*P* < 0.05, Fig. 10c). Similarly, the positive effects of hypoxia on EMT process were reversed by AGAP2-AS1 knockdown in Hep3B cells (*P* < 0.05, Fig. 10d). In conclusion, these results indicated that AGAP2-AS1 up-regulation functions in hypoxia-induced process on HCC cells.

**Fig. 10:** AGAP2-AS1 mediates the promoting effects of hypoxia on metastasis and EMT of HCC cells. **a** The expressions of HIF-1α in different time points in normoxia and hypoxia condition. **b** The levels of AGAP2-AS1 in Hep3B cells cultured in normoxia and hypoxia. **c** Transwell assays revealed that hypoxia promoted migration and invasion of Hep3B cells, while AGAP2-AS1 knockdown abolished the effects of hypoxia. **d** Hypoxia facilitated the EMT process of Hep3B cells and AGAP2-AS1 knockdown showed an opposite effect. *P < 0.05

RETRACTED

## Discussion

In recent years, lncRNAs profiling and functional assays of various types of cancers have provided accumulating evidence supporting the critical role of lncRNAs in tumor growth and progression [29]. LncRNAs have been proposed as novel diagnostic biomarkers, effective prognostic predictors and attractive therapeutic targets of HCC [30, 31]. In this study, we showed for the first time that lncRNA AGAP2-AS1 was significantly up-regulated in HCC tissues and cell lines. Moreover, the expression of AGAP2-AS1 was remarkably associated with the large size, metastatic, recurrent, and high histological grade phenotype of HCC (Additional file 6: Figure S6). These data strongly suggest that AGAP2-AS1 is an oncogene in HCC and plays a critical role in the progression of HCC.

Previous studies confirmed that lncRNA AGAP2-AS1 was identified as a diagnostic and prognosis marker in cancers [11, 13]. In this study, we demonstrated that AGAP2-AS1 promoted cell proliferation, migration, invasion, EMT progress and inhibited apoptosis by gain- and loss-of function experiment in vitro and in vivo. It has been reported that the aberrant lncRNAs act as ceRNAs for miRNAs to modulate tumor development and progression [15]. In this study, we confirmed miR-16-5p was obviously down-regulated and negatively correlated with AGAP2-AS1 in HCC tissues. On the other words, bioinformatics analysis, luciferase reporter assay, biotin pull-down assay and RIP assay all defined that miR-16-5p was a target of AGAP2-AS1 in HCC cells. And a reciprocal repression of AGAP2-AS1 and miR-16-5p was confirmed in HCC cells. Moreover, we demonstrated that miR-16-5p exerted its suppressive effects on proliferation, migration, invasion and EMT progress of HCC cells. Through the rescued experiment, our data suggest that miR-16-5p mediated the biological function of AGAP2-AS1 on HCC cells. To confirm that whether AGAP2-AS1 and miR-16-5p could serve as valuable biomarkers for diagnosis and prognostic prediction, we found both high AGAP2-AS1 or low miR-16-5p were significantly associated with poor clinical features of HCC patients. Furthermore, we confirmed that AGAP2-AS1 overexpression and miR-16-5p underexpression as well as their combination were obviously correlated with worse prognosis of HCC patients. These results suggest that AGAP2-AS1 and miR-16-5p may be promising predictors for the prognosis of HCC patients.

Annexin A11 (ANXA11), one of Annexins family of calcium (Ca^2+^)-regulated phospholipid-binding proteins, which are associated with cancer progression, metastasis, apoptosis, cell growth [32, 33]. Here, we confirmed that ANXA11 was a direct downstream target of miR-16-5p and mediated the biological function of miR-16-5p and AGAP2-AS1 in HCC. MiR-16-5p overexpression or knockdown accordingly altered the luciferase activity of wt 3’UTR but not mt 3’UTR of ANXA11. Moreover, miR-16-5p negatively regulated ANXA11 abundance in HCC cells. In addition, miR-16-5p was inversely correlated with the expressions of ANXA11 in HCC tissues. Restoration of ANXA11 expression reversed the effects of miR-16-5p and AGAP2-AS1 on HCC cells. The downstream of ANXA11, AKT phosphorylation, mediated the effects on cell proliferation, migration, invasion and apoptosis. Taken together, these results demonstrated that AGAP2-AS1 exert an oncogene role via miR-16-5p/ANXA11/AKT axis in HCC.

RETRACTED

Finally, hypoxia environment is a critical cause for HCC metastasis and leads to abnormal expression of lncRNAs [34]. Previous studies confirmed that miR-16-5p, the target of lncRNA AGAP2-AS1, was regulated in hypoxia condition. Therefore, we tried to explore the correlation between hypoxia and AGAP2-AS1 in HCC. Our data showed that AGAP2-AS1 was significantly increased in hypoxia. Moreover, AGAP2-AS1 knockdown abolished the promoting effects of hypoxia on migration, invasion and EMT process of HCC cells. These results suggest that hypoxia-induced AGAP2-AS1 overexpression promotes the metastasis and EMT of HCC.

In conclusion, we demonstrated that AGAP2-AS1 was up-regulated in HCC, and could promote cell proliferation, migration, invasion, EMT progression and inhibited apoptosis of HCC cells via AGAP2-AS1/miR-16-5p/ANXA11/AKT axis, which could be a valuable and promising therapeutic target for HCC.

## Conclusions

To conclude, our data offer the promising evidence that AGAP2-AS1 overexpression acts as an independent risk factor for indicating poor prognosis of HCC patients. AGAP2-AS1 facilitates HCC cell proliferation, migration, invasion, EMT progress and inhibited apoptosis in vitro and in vivo. miR-16-5p was identified as not only a target but also a functional mediator of AGAP2-AS1 in HCC cells. ANXA11 was a direct target gene of miR-16-5p and mediated its biological effects by AKT phosphorylation. In conclusion, AGAP2-AS1/miR-16-5p/ANXA11/AKT axis promoted cell growth and metastasis of HCC. This finding will improve understanding of mechanism involved in cancer progression and provide novel targets for the molecular treatment of HCC.

## Additional files

Additional file 1: **Figure S1**. Western blot analysis of EMT-related markers expression in the presence and absence of AGAP2-AS1. *n* = three independent experiments. *P < 0.05. (TIF 183 kb)

Additional file 2: **Figure S2**. The animal photos revealed that AGAP2-AS1 overexpression significantly promoted, while AGAP2-AS1 knockdown inhibited tumor growth in vivo*. (TIF 747 kb)*

Additional file 3: **Figure S3**. The pictures showed that overexpression of miR-16-5p inhibited cell proliferation (A), migration (B), invasion (c) and promoted apoptosis (d) in HCCLM3 cells, while down-regulation of miR-16-5p promoted cell proliferation (A), migration (b), invasion (c) and inhibited apoptosis (d) in Hep3B cells. (TIF 4145 kb)

Additional file 4: **Figure S4**. ANXA11 restoration abrogated the effects of miR-16-5p overexpression on cell proliferation (A), migration (B), invasion (c) and apoptosis (d) of HCCLM3 cells. ANXA11 knockdown reversed the promotive effects of miR-16-5p knockdown in Hep3B cells (a-d). (TIF 4265 kb)

Additional file 5: **Figure S5**. AKT inhibitor MK2206, or AKT phosphorylation activator IGF-1, abolished the cell proliferation (a), migration (b), invasion (c) and apoptosis (d) of HCC cells which were transduced of ANXA11 vectors. *P < 0.05. (TIF 4113 kb)

Additional file 6: **Figure S6**. A schematic diagram representing the role of AGAP2-AS1, functioning as a competitive endogenous RNA. (TIF 59 kb)

RETRACTED

## Abbreviations

3′-UTR: 3′-untranslated region
AFP: Alpha-fetoprotein
ANXA11: Annexin A11
EMT: Epithelial-mesenchymal transition
H&E: Hematoxylin and eosin
HCC: Hepatocellular carcinoma
IF: Immunofluorescence
IHC: Immunohistochemistry
lncRNA: Long non-coding RNA
miRNAs: microRNAs
qRT-PCR: Real-time quantitative reverse transcription polymerase chain reaction
RIP: RNA immunoprecipitation
TNM: Tumor-node-metastasis
